The article "ppENK Gene Methylation Status in the Development of Pancreatic Carcinoma" was published in 2013. Journal: Gastroenterol Res Pract.

# *ppENK* Gene Methylation Status in the Development of Pancreatic Carcinoma

**DOI:** 10.1155/2013/130927

**Published:** 2013-05-28

**Authors:** Lixin Yang, Hong Yang, Jingnan Li, Jianyu Hao, Jiaming Qian

**Affiliations:** ^1^Department of Gastroenterology, Beijing Chaoyang Hospital, Capital University of Medical Sciences, Beijing 100020, China; ^2^Department of Gastroenterology, Peking Union Medical College Hospital, Peking Union Medical College, Chinese Academy of Medical Science, Beijing 100730, China

## Abstract

*Objective*. To explore the association of hypermethylation of the proenkephalin gene (*ppENK*) with pancreatic carcinoma and to identify the effects of a demethylating agent on pancreatic cell lines. *Method*. Human pancreatic cancer tissues and five pancreatic carcinoma cell lines, as well as normal pancreatic tissue, were used. *ppENK* methylation status was detected by MS-PCR (methylation-specific PCR). *Results*. Methylation of *ppENK* was detected in 90.3% (28/31) of the human pancreatic carcinoma tissues but was not seen in normal pancreatic tissue. There was no correlation between the extent of methylation of *ppENK* and the clinicopathological features of the pancreatic carcinomas. Methylated *ppENK* was detected in all the pancreatic cancer cell lines and was associated with loss of mRNA expression in the pancreatic carcinoma cell lines and normal pancreatic tissue. After treatment with 5-aza-dC, methylated *ppENK* was not detected and the inhibition of *ppENK* mRNA expression was reversed. *Conclusions*. Inhibition of *ppENK* expression by a change in its methylation status plays an important role in pancreatic carcinogenesis. *ppENK* methylation is thus an important molecular event that distinguishes pancreatic carcinoma tissue from normal pancreatic tissue. Effects on cell growth, apoptosis, and the cell cycle may contribute to changes of *ppENK* methylation status.

## 1. Introduction

Pancreatic carcinoma is highly malignant and has a poor prognosis. The overall 5-year survival rate for pancreatic cancer does not exceed 5% in most studies, because it is generally diagnosed too late to allow surgery, which is still considered a curative treatment for pancreatic cancer. The incidence of pancreatic cancer has steadily increased in recent years. Its pathogenesis is not understood, and novel treatments are urgently needed [1].

The human *ppENK* gene has been localized to chromosome 8, at q23-q24, and consists of four transcribed exons and three introns. It is a neuropeptide transmitter gene and encodes Met-enkephalin, which is a topically active inhibitor of pancreatic cancers that interacts with the opioid growth factor receptor [2, 3].

The article "ppENK Gene Methylation Status in the Development of Pancreatic Carcinoma" was published in 2013. Journal: Gastroenterol Res Pract.

DNA methylation is an important regulator of gene transcription, and its role in carcinogenesis has been a topic of considerable interest in the last few years. Alterations in DNA methylation are common in a variety of tumors as well as in normal development. Of all the epigenetic mechanisms, hypermethylation, which represses transcription of tumor suppressor genes leading to gene silencing, has been the most extensively studied [4–6].

The aim of this study was to explore the association of hypermethylation of *ppENK* with pancreatic carcinoma and to examine the effects of a demethylating agent on pancreatic cell lines.

## 2. Materials and Methods

### 2.1. Cell Lines and Tissues

The human pancreatic carcinoma cell lines Panc-1, Pupan-1, Aspc-1, PC3, and SW1990 were obtained from the Peking Union Medical College Hospital. Thirty-two pancreata surgically resected at the Peking Union Medical College Hospital were selected. Normal pancreatic tissues were obtained from surgical resections at the Peking Union Medical College Hospital. The institutional review committee for clinical investigation reviewed and approved the collection of tissue samples for genetic analysis. Information on the following was available for all the selected cases: age, sex, diagnosis, CA19-9 levels, liver function (especially jaundice), tumor size, location, and clinical stage. Normal pancreatic tissue was taken from autopsy specimens. We examined the association of the methylation status of *ppENK* with tumor stage, size, location, sex, age, smoking, drinking, and so forth.

### 2.2. Microdissection of Tumor Cells and DNA Isolation

Two 20 *μ*m serial sections of formalin-fixed, paraffin-embedded tissue from 9 patients were deparaffinized with xylene for 30 minutes (the xylene was changed every 10 minutes) and dehydrated in an ethanol series. The slides were then stained with eosin to facilitate microdissection. Pancreatic ductal adenocarcinoma was identified under a microscope by a single pathologist, and the areas of interest were manually microdissected. An estimated 10% to 20% of the cells collected were surrounding nonductal cells. Nontumor tissue was collected in a separate tube. The microdissected tissues were transferred to a 1.5 mL microcentrifuge tube containing 50 *μ*L of 1x TK buffer (0.05 mmol/L Tris-HCl, pH 8.9; 2 mmol/L EDTA; 1 mmol/L NaCl; 0.5% Tween 20; and 0.2 mg/mL proteinase K) and incubated at 56°C overnight. The tubes were placed in a 100°C block for 10 minutes to inactivate proteinase K. Genomic DNA was extracted from 5 to 10 mg paraffin-embedded tissue using a Puregene DNA isolation kit following the protocol for DNA isolation provided. DNA was quantified by ultraviolet spectrophotometry and stored at 4°C.

The article "ppENK Gene Methylation Status in the Development of Pancreatic Carcinoma" was published in 2013. Journal: Gastroenterol Res Pract.

### 2.3. Reverse-Transcriptase Polymerase Chain Reaction (RT-PCR)

RNA from the pancreatic cancer cell lines was isolated with Trizol Reagent (Life Technologies, Rockville, MD, USA). Samples of each RNA were reverse-transcribed using a Superscript II kit (Life Technologies). PCR primers were 5′-CCG AAT GCA GCC AGG ATT G-3′ (sense) and 5′-GTG CTG GTG CCA TCT TGA G-3′ (antisense). A 179 bp PCR product was then amplified along with glyceraldehyde-3-phosphate dehydrogenase (GAPDH) in the following conditions: 95°C for 5 minutes; 35 cycles of amplification (95°C for 30 seconds, 60°C for 30 seconds, and 72°C for 300 seconds); 10 minutes at 72°C. The PCR reaction products were resolved by electrophoresis on 2% agarose gels and stained with ethidium bromide.

### 2.4. Methylation-Specific PCR (MSP)

*ppENK* methylation status was detected by MSP. Genomic DNA was isolated from the cell lines and frozen normal pancreatic samples using a tissue DNA isolation kit. Pancreatic carcinoma cells were microdissected from six paraffin-embedded blocks before DNA isolation. DNA was modified by sodium bisulfite as previously described [7].

The bisulfite treatment was performed on each dissected sample (50 *μ*L containing 500 to 10,000 cells) by incubating the DNA at 50°C for 16 hours, as previously described [8]. The modified DNA was purified using a Wizard DNA Clean-up System (Promega, Madison, WI, USA). After that, the polymerase chain reaction (PCR) was performed without ethanol precipitation so as to decrease the loss of DNA [9].

MSP was performed on samples of bisulfite-modified DNA using primers specific for unmethylated *ppENK *(sense: 5′-TTGTGTGGGGAGTTATTGAGT-3′; antisense: 5′-CACCTTCACAAAAAAAATCAATC-3′) or methylated *ppENK *(5′-TGTGGGGAGTTATCGAGC-3′ and 5′-GCCTTCGCGAAAAAAATCG-3′). The PCR product was then amplified along with glyceraldehyde-3-phosphate dehydrogenase (GAPDH) in the following conditions: 94°C for 13 minutes; 45 cycles of amplification (94°C for 30 seconds, 62°C for 30 seconds, and 72°C for 30 seconds); 3 minutes at 72°C. The PCR reaction products were resolved by electrophoresis on 2% agarose gels and stained with ethidium bromide.

### 2.5. 5-aza-dC

Cells of two pancreatic carcinoma cell lines (Panc-1, Aspc-1) were treated with a final concentration of 1.0 *μ*M of the demethylating agent 5-aza-dC (Sigma Chemical Co.); the Aspc-1 was treated for 96 h and the Panc-1 cells for 120 h. Cell growth was measured by the MTT method, and apoptosis and the phases of the cell cycle were analyzed by flow cytometry after PI staining. 

### 2.6. Statistical Analysis

Each experiment was repeated at least three times, and the experimental data are reported as means ± standard deviations. Statistical analysis was performed with the SPSS11.0 statistical software package. The chi-square analysis, *t*-test, Fisher's exact test, and calculated OR values were used; *P* < 0.05 indicated significant difference. Fisher's exact test was used to analyze the association of the methylation status of *ppENK* with tumor stage, size, location, sex, age, smoking, drinking, and so forth.

The article "ppENK Gene Methylation Status in the Development of Pancreatic Carcinoma" was published in 2013. Journal: Gastroenterol Res Pract.

## 3. Results

### 3.1. Pancreatic Cancer Tissue

*ppENK* was methylated in twenty-eight (90.3%) of the 31 samples of pancreatic cancer tissues, whereas it was not methylated in normal pancreatic tissue. There was no correlation between the extent of methylation of *ppENK* and clinicopathological features of the tumors. 

The size of the *ppENK* methylation target band (M band) is 96 bp (Figure 1).

### 3.2. The Relation between Extent of **ppENK ** Methylation and Clinicopathological Features of the Pancreatic Carcinomas

There was no correlation between the extent of methylation of *ppENK* and clinicopathological features of the pancreatic carcinomas such as tumor stage, size, location, sex, age, smoking, and drinking, (Table 1).

### 3.3. Pancreatic Carcinoma Cell Lines

In the five pancreatic carcinoma cell lines, methylated *ppENK* was demonstrated and no *ppENK* mRNA was detected. Methylated *ppENK* is associated with absence of *ppENK* mRNA expression. 

### 3.4. **ppENK ** Gene mRNA Expression in Pancreatic Cancer Cell Lines

We examined expression of *ppENK *using RT-PCR in the 5 pancreatic cell lines. *ppENK* mRNA was detected in normal pancreatic tissue but not in the five pancreatic carcinoma cell lines (Panc-1, Pupan-1, Aspc-1, PC3, and SW1990) (Figure 2).

### 3.5. Analysis of **ppENK ** Gene Methylation in Pancreatic Cancer Cell Lines

DNA was extracted from the five pancreatic cancer cell lines (Panc-1, PC3, Pu-Pan-1, SW1990, and Aspc-1), modified by sulfite and amplified by MS-PCR. The results showed that the target band (M band) could be seen in the five pancreatic cancer cell lines. Thus methylated *ppENK* was detected in all five pancreatic cancer cell lines. Methylated *ppENK* is associated with the absence of* ppENK* mRNA expression in pancreatic carcinoma cell lines and normal pancreatic tissue (*P* = 0.018) (Figure 3).

### 3.6. The Effect of the Demethylating Agent 5-aza-dC on Pancreatic Cancer Cell Proliferation

Based on the MS-PCR results and the origins of the pancreatic cancer cell lines, we chose the Panc-1 and Aspc-1 to test the effect of 5-aza-dC on proliferation. Samples of 10^3^ cells of the two cell lines (Panc-1 and Aspc-1) were seeded in 96 well plates, cultured 1–5 days, and cell numbers were determined using the MTT assay. The proliferation of Aspc-1 decreased significantly (1.608 ± 0.219) in response to 5-aza-dC (1.0 *μ*M) at 96 h (control: 2.644 ± 0.247) and a similar effect could be seen in Panc-1 at 120 h (Tables 2 and 3; Figures 4 and 5).

The article "ppENK Gene Methylation Status in the Development of Pancreatic Carcinoma" was published in 2013. Journal: Gastroenterol Res Pract.

### 3.7. The Effect of the Demethylating Agent 5-aza-dC on Apoptosis and the Cell Cycle of the Pancreatic Cancer Cell Lines Panc-1 and Aspc-1

Flow analysis was used to assess the cell cycle of cells. For flow analysis, Panc-1 and Aspc-1 were stained with propidium iodide (PI, Sigma) as described and were used to estimate proportions of cells in the G1/S and G2/M phases of the cell cycle. The frequencies of apoptosis of of Panc-1 and Aspc-1 induced by 5-aza-dC (1.0 *μ*M) were 31.57 ± 6.76% and 16.6 ± 8.22%. In the absence of 5-aza-dC the frequencies were 3.21 ± 1.43%, 3.82 ± 1.71%. The frequency of cells in G1 phase was increased concomitant with a decrease in the percentage of S phase cells in Panc-1 (*P* < 0.05) but not in Aspc-1. 

### 3.8. The Percentage of Apoptosis Detected by Flow Cytometry (PI Staining)

After treatment with 1 *μ*M 5-aza-dC for 5 days, Panc-1 cells were stained with PI and apoptosis was detected by flow cytometry. The average apoptosis percentage was 31.57 ± 6.76% in the treatment group, higher than the control group (3.21 ± 1.43%, *P* < 0.05). The average apoptosis percentage of Aspc-1 cells was 31.57 ± 6.76% in the treatment group and 3.82 ± 1.71% in the control group; the percentage apoptosis increased after treatment, but the effect in this case was not statistically significant (*P* > 0.05) (Figures 6 and 7; Table 4).

### 3.9. Cell Cycle Distribution Detected by Flow Cytometry

Compared with the control group, the proportion of G1 phase Panc-1 cells was significantly increased in the treatment group, and the proportion in the DNA synthesis phase (S phase) was significantly reduced (*P* < 0.05), but in the Aspc-1 cells there was no noticeable increase in G1 phase or decrease in S phase (Tables 5 and 6; Figure 8).

### 3.10. Effect of the Demethylating Agent 5-aza-dC on **ppENK ** Gene Expression

After treatment of the 2 pancreatic carcinoma cell lines with 5-aza-dC, *ppENK* mRNA expression was reversed. The 180 bp target band was detected in the treatment group and the normal pancreas but not in the control group, while the internal reference using GAPDH could be seen (Figure 9).

Compared with the control group using FluorChem (data analysis software), *ppENK* gene expression in Panc-1 and AspC-1 cells was significantly increased in the treatment group (*P* < 0.05). The results show that 5-aza-dC can reverse the inhibition of *ppENK* gene expression.

The article "ppENK Gene Methylation Status in the Development of Pancreatic Carcinoma" was published in 2013. Journal: Gastroenterol Res Pract.

### 3.11. Effects of the Demethylating Agent 5-aza-dC on Panc-1 and Aspc-1 Cell Methylation

After treatment with the demethylating agent 5-aza-dC, extraction of cell DNA and modification by sulfite, MS-PCR, failed to detect the *ppENK* methylation target band (Figure 10).

## 4. Discussion

The *ppENK* gene encodes met-enkephalin, which is a tonically active inhibitory factor that interacts with the opioid growth factor receptor. Zagon and McLaughlin reported that met-enkephalin inhibited the growth of several human tumors including pancreatic cancers [3]. Comb et al. reported that methylation of CpG islands within the *ppENK* gene inhibited its expression by directly interfering with the binding of a positively acting transcription factor [2]. Therefore, methylation of *ppENK* during pancreatic carcinogenesis may promote cell growth. Here, our aim was to explore the association between hypermethylation of *ppENK* and pancreatic carcinoma and to study the effects of a demethylating agent on pancreatic cell lines.

*ppENK* methylation was confirmed in 90.3% (28 out of 31) of the examined samples of pancreatic cancer tissue, but there was no association between methylation and clinicopathological features. Additionally, methylated *ppENK* was detected in five pancreatic carcinoma cell lines (SW1990, Panc-1, PC3, Aspc-1, and Pupan-1) that showed no expression of *ppENK* mRNA, which corroborates the findings of previous studies. Overall, these results confirm that silencing of the* ppENK* gene due to methylation may be an important event in carcinogenesis and the development of pancreatic cancer. However, animal studies and clinical research are warranted to validate this view.

There are several methods of detecting methylation, and each has its own advantages and a range of applications. Currently the most widely used technique is sodium bisulfite modification of DNA and subsequent methylation-specific PCR 10 (MSP), also used in our study. Using two pairs of highly specific primers, this method is able to amplify specific target sequences and distinguish a methylated template from a nonmethylated background with high sensitivity. In fact, as the most sensitive method of detecting methylation, MSP can be effectively used to analyze paraffin specimens, as well as to trace samples such as blood or stool. Therefore, MSP appears to be a useful method for early diagnosis of pancreatic cancer [8, 10–12]. It should be noted, however, that although tumor cell lines are free of the contamination with normal cells otherwise associated with in vivo samples, and they preserve the molecular abnormalities of the tumors and the malignant phenotype, their biological characteristics may change after long-term cultivation. Hence, in vitro and in vivo results should be interpreted together.

The article "ppENK Gene Methylation Status in the Development of Pancreatic Carcinoma" was published in 2013. Journal: Gastroenterol Res Pract.

Two of the five pancreatic cancer cell lines, Panc-1 and PC3, were derived from primary tumors in earlier clinical stages, while Aspc-1, SW1990, and Pupan-1 were derived from metastatic tumors in later clinical stages. We therefore selected Aspc-1 and Panc-1 for the purposes of this study. Cell proliferation was found to decrease with increasing dose of 5-aza-dC (0.4–1.0 *μ*M), confirming that 5-aza-dC inhibits the growth of pancreatic cancer cells. There was no significant difference between the responses of the two cell lines at a concentration of 1.0 *μ*M 5-aza-dC (*t* = −0.049, *P* = 0.962).

Apoptosis is an important aspect of the balance between cell division and cell loss. It plays a role in many diseases such as cancer and autoimmune disorders, among others. The results of PI staining and flow cytometry of the Panc-1 and Aspc-1 cell lines in our study showed that apoptosis was triggered by different levels of 5-aza-dC in these two types of cells. Treatment with the demethylating agent resulted in a significantly higher rate of apoptosis in Panc-1 cells than in untreated controls (*P* < 0.05). In Aspc-1 cells, apoptosis increased from 3.82 ± 1.71% to 16.6 ± 8.22% after treatment, but this effect was not statistically significant (*P* = 0.058), possibly due to the small sample size.

The malignant phenotype of tumor cells depends, to a substantial extent, on the rate of cell proliferation, which in turn depends on the duration of the cell cycle and on the ratio of cell proliferation to cell death. Thus, in addition to measuring the rate of apoptosis, we should also be interested in any change to the phases of the cell cycle and the proportion of tumor cells that are involved. In our study, Panc-1 cells treated with 5-aza-dC had a longer G1 phase and a correspondingly shorter S phase than untreated controls (*P* < 0.05). While the same trend was observed in the Aspc-1 cell line, it did not reach statistical significance. It is, therefore, possible that 5-aza-dC could have a different impact on different types of tumor cells, or it could affect different phases of the division cycle. This hypothesis requires further study [13].

In line with previous studies, our findings showed that 5-aza-dC treatment reversed the expression of *ppENK* mRNA in the pancreatic cancer cell lines Panc-1 and Aspc-1, though to varying degrees (*P* < 0.05). *ppENK* methylation could be seen before the treatment, but after treatment it was below detection levels. However, the nonmethylated primers failed to amplify the target band (U band), suggesting that the amount of 5-aza-dC used in the experiment may not have been enough to achieve complete demethylation. MSP assay primers are typically designed based on all CpG sites within a CpG island, but, in fact, not all CpG sites are fully methylated or unmethylated. Because of this inconsistency, it may be difficult to amplify target fragments, and increasing the levels of 5-aza-dC may yield clearer results. Overall, our study provides more evidence that the *ppENK* gene is inactivated due to methylation and that changes in methylation status may promote cell apoptosis and inhibit the proliferation of pancreatic cancer cells [14–16].

The article "ppENK Gene Methylation Status in the Development of Pancreatic Carcinoma" was published in 2013. Journal: Gastroenterol Res Pract.

In conclusion, we show that *ppENK* inactivation due to changes in methylation plays an important role in pancreatic carcinogenesis. *ppENK* methylation is an important molecular event that could help to distinguish pancreatic carcinoma from normal tissue. Methylation of *ppENK* may also be affected by cell growth, cell apoptosis, and the duration of the cell cycle.

## Figures and Tables

**Figure 1:** MSP of *ppENK* CpG islands. A visible PCR product in lane U indicates the presence of unmethylated gene promoters; the presence of product in lane M indicates the presence of promoter methylation.

**Figure 2:** RT-PCR analysis of 5 pancreatic carcinoma cell lines. The *ppENK* PCR band is 179 bp. Glyceraldehyde-3-phosphate dehydrogenase (GAPDH) serves as an RNA control: lane 1, normal pancreatic tissue (frozen tissue); lane 2, Panc-1; lane 3, Pupan-1; lane 4, SW1990; lane 5, PC3; lane 1, Aspc-1.

**Figure 3:** The results of MSP of *ppENK* CpG islands. A visible PCR product in lane U indicates the presence of unmethylated gene promoters; the presence of product in lane M indicates the presence of promoter methylation. *ppENK*: lane 1, Aspc-1; lane 2, Panc-1; lane 3, Pupan-1; lane 4, SW1990; lane 5, PC3.

**Figure 4:** MTT analysis of Aspc-1.

**Figure 5:** MTT analysis of Panc-1.

**Figure 6:** Comparison of apoptotic rates. Aspc-1, Panc-1 control; Aspc-1+, Panc-1+ treatment.

**Figure 7:** (a) Panc-1 control. (b) Panc-1 treatment. (c) Aspc-1 control. (d) Aspc-1 treatment.

**Figure 8:** (a) Panc-1 control. (b) Panc-1 treatment. (c) Aspc-1 control. (d) Aspc-1 treatment.

**Figure 9:** RT-PCR analysis of the 5 pancreatic carcinoma cell lines. Glyceraldehyde-3-phosphate dehydrogenase (GAPDH) serves as an RNA control. The two cancer cell lines do not express *ppENK*. Treatment of Aspc-1 and Panc-1 with 5-aza-2-deoxycytidine restores the expression of *ppENK*: lane 1, normal pancreatic tissue (frozen tissue); lane 2, Aspc-1 (before the treatment); lane 3, Aspc-1 (after); lane 4, Panc-1 (before); lane 5, Panc-1 (after); lane 6, negative control.

The article "ppENK Gene Methylation Status in the Development of Pancreatic Carcinoma" was published in 2013. Journal: Gastroenterol Res Pract.

**Figure 10:** The results of MSP of *ppENK* CpG islands after treatment with 5-aza-2-deoxycytidine. A visible PCR product in lane U indicates the presence of unmethylated gene promoters; the presence of product in lane M indicates the presence of promoter methylation. *ppENK:* lane 1, Aspc-1; lane 2, Panc-1; lane 3, pancreatic carcinoma tissue.

**Table 1:** Case characteristics.

	Case	*ppENK * methylation	*ppENK * nonmethylation	Fisher's exact test
Differentiation	31	28	3	*P* = 0.125
Poor	8	6	2	
Moderate	15	15	0	
High	8	7	1	

Tumor stage	31	28	3	*P* = 0.533; OR = 1.556
I/II	21	18	3	
III/IV	10	10	0	

Tumor size	29	27	2	*P* = 1.000; OR = 1.455
≤3 cm	12	11	1	
>3 cm	17	16	1	

Tumor location	31	28	3	*P* = 1.000; OR = 0.947
Head	21	19	2	
Body and tail	10	9	1	

Sex	31	28	3	*P* = 1.000; OR = 1.217
M	26	23	3	
F	5	5	0	

Age	31	28	3	*P* = 1.000; OR = 1.733
>60 years	17	15	2	
≤60 years	14	13	1	

Smoking	31	28	3	*P* = 0.205; OR = 0.800
No	22	20	2	
Yes	9	8	1	

Alcohol	31	28	3	*P* = 0.271; OR = 0.154
No	28	26	2	
Yes	3	2	1	

CA199	27	24	3	*P* = 0.545; OR = 0.526
>37 u/mL	21	19	2	
<37 u/mL	6	5	1	

OR: odds ratio.

**Table 2:** MTT analysis of Aspc-1.

	Control	0.4 *µ*M	0.6 *µ*M	0.8 *µ*M	1.0 *µ*M
24 h	1.100 ± 0.050	1.095 ± 0.100	1.073 ± 0.132	0.998 ± 0.218	0.932 ± 0.066
48 h	1.783 ± 0.211	1.567 ± 0.181	1.463 ± 0.106	1.458 ± 0.205	1.365 ± 0.127
72 h	2.521 ± 0.069	2.346 ± 0.145	2.271 ± 0.094	1.872 ± 0.345*	1.598 ± 0.165*
96 h	2.644 ± 0.247	2.269 ± 0.266	1.953 ± 0.243*	1.723 ± 0.186*	1.608 ± 0.219*
120 h	2.964 ± 0.184	2.799 ± 0.222	2.322 ± 0.284*	2.326 ± 0.257*	1.978 ± 0.244*

*P < 0.05 versus control OD.

**Table 3:** MTT analysis of Panc-1.

	Control	0.4 *µ*M	0.6 *µ*M	0.8 *µ*M	1.0 *µ*M
24 h	1.193 ± 0.1811	0.905 ± 0.201	0.764 ± 0.164	0.792 ± 0.176	0.770 ± 0.068
48 h	1.740 ± 0.146	1.591 ± 0.090	1.458 ± 0.099	1.437 ± 0.162	1.414 ± 0128
72 h	2.422 ± 0.168	2.201 ± 0.186	1.812 ± 0.181*	1.533 ± 0.125*	1.479 ± 0.121*
96 h	2.754 ± 0.059	2.451 ± 0.226	1.966 ± 0.215	1.786 ± 0.164*	1.515 ± 0.184*
120 h	2.934 ± 0.071	2.503 ± 0.047*	2.215 ± 0.080*	1.916 ± 0.137*	1.734 ± 0.050*

*P < 0.05 versus control OD.

**Table 4:** Comparison of apoptotic rates.

Cell	Treatment (*X* ± *S*%)	Control (*X* ± *S*%)	*P *
Aspc-1	16.6 ± 8.22	3.82 ± 1.71	0.058
Panc-1	31.57 ± 6.76	3.21 ± 1.43*	0.002

*P <  0.05, treatment versus control; *n* = 3.

**Table 5:** The cell cycle of Panc-1.

Phase	Treatment (*X* ± *S*%)	Control (*X* ± *S*%)	*P *
G1 phase	67.87 ± 2.72	54.57 ± 7.18*	0.040
S phase	22.37 ± 4.31	33.73 ± 4.63*	0.036

*P < 0.05, Aspc-1 versus control; *n* = 3.

**Table 6:** The cell cycle of Aspc-1.

Phase	Treatment (*X* ± *S*%)	Control (*X* ± *S*%)	*P *
G1 phase	61.20 ± 10.35	52.43 ± 3.46	0.236
S phase	27.27 ± 5.67	35.20 ± 0.85	0.075

*P < 0.05, Aspc-1 versus control; *n* = 3.
